# Transplantation of Mouse Induced Pluripotent Stem Cell-Derived Podocytes in a Mouse Model of Membranous Nephropathy Attenuates Proteinuria

This article has been retracted.

**DOI:** 10.1038/s41598-019-51770-0

**Published:** 2019-10-29

**Authors:** Amin Ahmadi, Reza Moghadasali, Vahid Ezzatizadeh, Zeinab Taghizadeh, Seyed Mahdi Nassiri, Mohammad Hassan Asghari-Vostikolaee, Mehdi Alikhani, Fatemeh Hadi, Reza Rahbarghazi, Reza Salman Yazdi, Hossein Baharvand, Nasser Aghdami

**Affiliations:** 1 Department of Stem Cells and Developmental Biology, Cell Science Research Center, Royan Institute for Stem Cell Biology and Technology, ACECR, Tehran, Iran; 2 Medical Genetics Department, Medical Laboratory Center, Royesh Medical Group, Tehran, Iran; 3 Department of Clinical Pathology, Faculty of Veterinary Medicine, University of Tehran, Tehran, Iran; 4 Animal Core Facility, Reproductive Biomedicine Research Center, Royan Institute for Biotechnology, ACECR, Tehran, Iran; 5 Department of Brain and Cognitive Sciences, Cell Science Research Center, Royan Institute for Stem Cell Biology and Technology, ACECR, Tehran, Iran; 6 Stem Cell Research Center, Tabriz University of Medical Sciences, Tabriz, Iran; 7 Department of Andrology, Reproductive Biomedicine Research Center, Royan Institute for Reproductive Biomedicine, ACECR, Tehran, Iran; 8 Department of Developmental Biology, University of Science and Culture, Tehran, Iran; 9 Department of Regenerative Medicine, Cell Science Research Center, Royan Institute for Stem Cell Biology and Technology, ACECR, Tehran, Iran

**Keywords:** Regeneration, Stem-cell differentiation, Induced pluripotent stem cells

## Abstract

Injury to podocytes is a principle cause of initiation and progression of both immune and non-immune mediated glomerular diseases that result in proteinuria and decreased function of the kidney. Current advances in regenerative medicine shed light on the therapeutic potential of cell-based strategies for treatment of such disorders. Thus, there is hope that generation and transplantation of podocytes from induced pluripotent stem cells (iPSCs), could potentially be used as a curative treatment for glomerulonephritis caused by podocytes injury and loss. Despite several reports on the generation of iPSC-derived podocytes, there are rare reports about successful use of these cells in animal models. In this study, we first generated a model of anti-podocyte antibody-induced heavy proteinuria that resembled human membranous nephropathy and was characterized by the presence of sub-epithelial immune deposits and podocytes loss. Thereafter, we showed that transplantation of functional iPSC-derived podocytes following podocytes depletion results in recruitment of iPSC-derived podocytes within the damaged glomerulus, and leads to attenuation of proteinuria and histological alterations. These results provided evidence that application of iPSCs-derived renal cells could be a possible therapeutic strategy to favorably influence glomerular diseases outcomes.

## Introduction

Nephrotic syndrome (NS), as a hallmark of glomerular disease (GD), is characterized by severe proteinuria (≥3.5 gr/d), edema, hypoalbuminemia, and various levels of hyperlipidemia^1^. There is a clear clinical correlation between proteinuria and subepithelial immune deposition in glomerular diseases that lead to nephrotic syndrome. Immune-mediated proteinuria has thus far been proposed to be induced by two different mechanisms including unspecific accumulation of immunoglobins (Igs) in glomerular capillary (i.e. membranoproliferative glomerulonephritis and systemic lupus nephritis) or binding of specific Igs to podocytes-associated targets leading to disruption and loss of podocytes (i.e. membranous nephropathy)^2,3^. Podocytes are highly specialized cells with a complex cytoarchitecture. They are composed of tertiary foot processes (FPs), as a major component of the glomerular filtration barrier. An exclusive intracellular junction, known as the slit diaphragm (SD), is responsible for FPs connections, serving as an ultimate barrier to regulate passage of macromolecules from the blood. Alterations of the unique actin-based morphology of FPs are a common feature of kidney disease^4^. Membranous nephropathy (MN), as one of the most common form of GDs causes NS and subsequently, end-stage renal disease in Caucasian adults, and is a form of immune-mediated glomerular injury characterized by subepithelial deposition of immune complexes, glomerular accumulation of IgG, C3, and C5b-9, and extensive FPs effacement^1,5^.

In contrast to the regenerative ability of tubular epithelial cells^6^, replacement of damaged podocytes remains a challenge^7^. As long as the rate of podocyte loss is limited, recuperation or repair of these cells is possible. Using animal models, it was shown that podocytes depletion of up to 20% can be compensated, most likely through induction of hypertrophy in the adjacent podocytes^8^. By contrast, a 20–40% loss of the podocytes can cause a scarring response and an over 50% loss of podocytes results in dysfunction of glomeruli filtration. These levels of podocytes depletion are accompanied by corresponding degrees of proteinuria due to the increased proportion of the involved glomeruli and remarkable reductions in renal clearance, as seen in immune-mediated NS^9–11^. Currently, therapeutic protocols for MN are often non-specific^12^ and rely on suppression of the immune system^13,14^.

According to recent reports, stem cell-based therapy could potentially be a novel therapeutic approach for chronic kidney diseases (CKD)^15–18^. Hence, there are reports on human/mouse iPSCs differentiation into podocytes^19–24^ and use of these cells *in vitro*^23,25^ or *in vivo*^26^. In addition, a recent study reported the beneficial effects of multilineage-differentiating stress-enduring (Muse) cells in an animal model of focal segmental glomerular sclerosis^27^. However, the ability of transplanted iPSC-podocytes to restore kidney function and structure in animal models of immune-mediated NS, remains to be studied.

In this study, following anti-podocyte antibody (APA) production, we generated a model of APA-induced heavy proteinuria that resembled human MN and was characterized by the presence of subepithelial immune deposits and podocytes loss. Thereafter, iPSCs from a mouse with proteinuria, were differentiated into podocytes that showed protein marker localization and functional characteristics of podocytes. The data revealed that iPSC-podocyte transplantation (PT) decreased proteinuria and improved histopathological features possibly through replacing lost podocytes.

## Results

### Generation, purification and characterization of anti-podocyte antibody (APA)

In this experiment, rabbits were immunized with a whole podocyte preparation. Following removal of the blood clot, rabbit anti-podocyte serum was collected, concentrated and complement-inactivated. Then, IgGs were isolated from the serum samples (Supplementary Fig. S1A).

SDS-PAGE analysis of the rabbit anti-mouse IgG showed 2 distinct bands with molecular weights of ~50 and ~25 kDa, indicative of rabbit IgG heavy and light chains, respectively (Supplementary Fig. S1B). Indirect ELISA titration of anti-podocyte IgG showed robust immunoreactivity of the antibody against the differentiated immortalized podocytes, which confirmed its functionality after purification (Supplementary Fig. S1C). Subsequently, immunofluorescence staining revealed specific surface and perinuclear cytoplasmic binding of the purified antibody to podocytes compared to the control (Supplementary Fig. S1D,E). In contrast, no binding in mesangial cells after incubation with APA or preimmune antibody was observed (PI; Supplementary Fig. S1F,G). Flow cytometric analysis results indicated that APA was bound to approximately 95% of the podocyte population (Supplementary Fig. S1H) with no remarkable interactions for APA in mesangial cells (Supplementary Fig. S1I) nor for PI in podocytes and mesangial cells (Supplementary Fig. S1K,L). In addition, no reaction to the isotopic control was observed in the podocyte and mesangial cells (Supplementary Fig. S1J,M). Specific fluorescence could be detected with APA, even at 1:1000 dilution. According to the Bradford assay, the concentration of purified IgG was 7.5 mg/ml.

### Generation and characterization of iPSCs from a mouse model of membranous nephropathy

Resemblance of the representative tail-tip fibroblast (TTFs; Supplementary Fig. S2A)- derived iPSCs to generally approved ESC lines, was verified in terms of morphology (Supplementary Fig. S2B); karyotype analysis (Supplementary Fig. S2C); teratoma formation (Supplementary Fig. S2D); and the presence of cells and structures presenting the 3 germ layers within the teratoma (Supplementary Fig. S2E–G); embryoid body (EB) formation (Supplementary Fig. S2H); and alkaline phosphatase expression (Supplementary Fig. S2I). Observations by fluorescence and immunofluorescence microscopy also confirmed the appropriate localization of green fluorescent protein (GFP) in the iPSCs (Supplementary Fig. S2J) and the presence of 4 pluripotency markers (Supplementary Fig. S2K–N) following long-term culture (passages 30–35), respectively.

### Differentiation and characterization of podocytes from iPSCs

Figure 1A depicts the protocol we used for differentiation of mouse iPSCs. First, GFP^+^ iPSC differentiation into nephrogenic intermediate mesoderm (NIM) was induced through formation of EBs (Supplementary Fig. S3A,B,I,J) followed by a culture of EBs. Previous studies that investigated renal differentiation of pluripotent cells relied on *Osr1*, *Pax2*, *Lhx1*, *Wt1*, *Eya1*, and *Sall1* as definitive markers for NIM formation^22,28–31^. According to this evidence, we analyzed their expressions at gene or protein levels. Immunofluorescence staining and quantitative reverse transcription polymerase chain reaction (qRT-PCR) analysis of NIM cells (Supplementary Fig. S3C) showed the expression of Osr1, a key upstream molecule in renal development, and Pax2 and Sall1^32,33^ at the protein levels (Fig. 1B). These cells also expressed *Lhx1*, *Eya*1, and *Wt1* at the transcriptional levels. Conversely, we observed downregulation of the pluripotency marker *Oct4* that occurred from the undifferentiated state to day 8 of differentiation (Fig. 1C). Following culture of NIM cells in basal medium that contained 15 ng/ml BMP7, 1 U/ml LIF, and 150 ng/ml glial cell line-derived neurotrophic factor (GDNF), we observed that the transcription levels of NPC marker genes *Six2, Hoxd11, Cited1, Sall1, Eya1, Pax2*, and *Wt1*^34^, up-regulated after day 3 of treatment (Fig. 1D). Key markers of NPCs namely, Six2, Pax2, and Wt1, were detected in iPSC-derived NPCs by immunostaining (Fig. 1E). The proportion of cells that expressed Wt1 and Pax2 increased on day 15 of induction together with expression of podocin as a podocyte marker (Fig. 1F) that represented podocyte progenitors^35^. The transcription levels of other podocyte marker genes such as *Synpo*, *Nphs1*, *Cd2ap*, and *Pdxl*, also up-regulated at the same time (Fig. 1G). Interestingly, transcription levels of *Nphs1*^19^ and *Pdxl*^36^ were comparable to those observed for iPSCs.

**Figure 1:** Generation and characterization of podocytes from induced pluripotent stem cells (iPSCs). (**A**) Experimental design and optimization of induced pluripotent stem cell (iPSCs) differentiation into podocytes. (**B**) Immunostaining for nephrogenic intermediate mesoderm (NIM) markers Osr1, Pax2 and Sall1 on day 8. Quantitative RT-PCR analyses of marker gene expression for (**C**) NIM and (**D**) NPC cells differentiated from iPSCs on days 8 and 12, respectively. Immunofluorescence analysis of (**E**) NPC and (**F**) podocyte progenitor markers. (**G**) Gene expression analysis confirmed the commitment to the podocyte fate by the increase in podocyte markers. (**H**) Immunofluorescence analysis for the podocyte marker proteins podocin, podocalyxin, synaptopodin, Wt1, and nephrin displayed a final induction towards green fluorescent protein (GFP)^+^ mature podocyte cells at passage 6. We also observed the presence of highly organized actin fibers within the podocyte cytoplasm. Immunostaining of iPSC-podocytes with the produced anti-podocyte antibody (APA) showed high immunoreactivity with these cells. (**I**) Scanning electron microscopy of iPSC-podocytes demonstrated a main cell body and (**J**) tight junction-like structures that were connected to the adjacent cells (arrows). (**K**) Cytoplasmic projections that extended from the cell body (arrows) and (**L**) tertiary projections at the end of processes of the cytoplasmic projections (arrows). (**M**) Doubling time graph for proliferative differentiated podocytes from iPSCs. (**N**) Quantitative RT-PCR analyses showed decreased expression levels of *Pax2* and increased expression levels for *Wt1, Synpo, Nphs2*, *Nphs1*, and *Pdxl* with increasing culture time. (**O**) Flow cytometry for podocin in iPSC-podocytes on day 22. Samples treated only with secondary antibodies were used as controls (red). Relative gene expression was normalized against *GAPDH*. The fold-change values are represented by mean ± SEM (n = 3). Scale bars: B, E, F, and H: 100 µm.

Overall, the cell progeny consisted of uniformly unspecialized and immature criteria with a large, rounded, and often binucleated phenotype (Supplementary Fig. S3D). Most cells differentiated into stretched or multi-angled cells on day 15 (Supplementary Fig. S3E,K). Following cell culture in VRAD + dexamethasone, the proliferative cells were sub-passaged and cultured in Roswell Park Memorial Institute (RPMI)−1640 medium where they developed into large cells that had a typical arborized pattern of foot process extensions (Supplementary Fig. S3F, G,L). The morphology of the latter cells was comparable to immortalized mouse podocytes incubated under non-permissive conditions that displayed characteristics of mature podocytes (Supplementary Fig. S3H).

As shown in Fig. 1H, immunostaining of the iPSC-podocytes showed that podocin, podocalyxin, synaptopodin, and nephrin proteins were localized within the cytoplasm of the cell body, the extensions, or the filamentous arrangement of the iPSC-podocytes. We performed phalloidin staining for filamentous actin (F-actin). F-actin is a filamentous protein that forms the contractile cytoskeleton which is considered to be a key component of podocytes and is necessary for proper glomerular filtration. The results showed the presence of highly organized actin fibers within the podocyte cytoplasm. Despite the expression of both Pax2 and Wt1 in the progenitors, only Wt1 was expressed in sub-passaged podocytes at the protein level. The iPSC-podocytes were also validated by immunostaining using previously generated APA. GFP was detected mainly in the nuclei of the majority of cells because we did not attach any localization signal to GFP when generating GFP^+^ iPS cells.

Analysis of scanning electron microscopy images showed that iPSC-podocyte had a typical arborized phenotype that consisted of a main cell body with elongated processes which extended to the periphery of the cells (Fig. 1I). There were tight junction-like structures between adjacent cells (Fig. 1J) and secondary as well as tertiary cytoplasmic processes that were projected from the cell bodies (Fig. 1K,L).

Although the iPSC-podocytes could proliferate, we observed growth arrest during passage 6, which confirmed that these podocytes behaved like mature podocytes at this stage (Fig. 1M). qRT-PCR analysis of mRNA expression showed up-regulation of *Wt1*, *Synpo*, *Nphs2*, *Nphs1*, and *Pdxl* with increased culture time or passage number. On the other hand, the expression levels of *Pax2* decreased (Fig. 1N).

Flow cytometry analysis for podocin revealed an average of 80% efficiency for this differentiation protocol (Fig. 1O).

### Functional traits of iPSC-podocytes

Podocytes and their cytoplasmic extensions develop an actin-based contractile system that contracts in response to insulin^37^ and angiotensin II (AII)^19,22^. We used immunofluorescence and phase-contrast microscopy to film a time-lapse recording of the dynamic changes in cell morphology. Our data showed that addition of 100 nM of insulin and 500 nM of AII induced contractions in the iPSC-podocyte cell body and shortened cytoplasmic processes (Supplementary Fig. S4A and Movie S1). A permeability assay was performed to assess the endocytic uptake of albumin as further evidence for the functional characteristics of the iPSC-podocytes^22,38^. Fluorescence microscopy observation of the Texas Red-labelled albumin showed accumulation of vesicles within the cytoplasm near the perinuclear region (Supplementary Fig. S4B).

### Therapeutic effect of iPSC-Podocytes on renal function in mice with anti-podocyte antibody (APA) induced proteinuria

A preliminary experiment of the administered doses showed that APA 2.8 mg/mouse results in initial proteinuria on day 5 that increased to maximum values on days 10–15. Despite a slight reduction within the next 20 days, the proteinuria remained stable until day 60. In addition, albumin content was quantified and corrected for urine creatinine. The urine albumin/creatinine ratio significantly increased to a maximum value on day 15. The control groups consisted of non-treated (NT) mice, whereas the PI groups consisted of mice that received 2.8 mg/mouse of normal rabbit IgG. There was no significant difference in renal functional between the control and PI-treated groups (Fig. 2B–J). Therefore, we used the PI groups as control groups for statistical analyses.

**Figure 2:** Analysis of serum and urine indices in anti-podocyte antibody (APA) treated and iPSC-podocyte transplanted mice. (**A**) Timeline of pre-immunization and antibody infusion in mice. Asterisks and hashtags indicate days on which specimens for urine, serum, and histology were obtained. (**B**–**J**) Quantification of Upro, Ualb/crea ratio, Stpro, Salb, BUN, Stg, Scho, Uur, and Scr in non-treated (●, NT), preimmune (■, PI), anti-podocyte nephropathy + phosphate-buffered saline (▲, APN + PBS), and APN + podocyte transplantation (▼, APN + PT) mice groups (n = 5) on the indicated days. (**K**) Serum third complement component (C3) levels in PI and anti-podocyte antibody (APA) treated mice on days 10 and 15 (n = 3). (**L**) Protein staining of SDS-PAGE gel loaded with 2.5 µl of urine samples collected on the indicated days in the PI, APN + PBS, and APN + PT groups. (**M**) Left panel: Western blots of urine from day10 probed for mouse IgG (IgG), albumin (alb), podocin (pod), and podocalyxin (pdx). Right panel: Western blots of urine probed for pdx and green fluorescent protein (GFP), 25 days after cell transplantation. The grouping of blots was cropped from different parts of one gel and exposures are made explicit. Values are expressed as mean ± SEM. PI vs. APN + PBS groups: a: p < 0.05, b: p < 0.01, and c: p < 0.001. APN + PBS vs. APN + PT groups: A’: p < 0.05, B’: p < 0.01, and C’: p < 0.001.

Evaluation of complementary system interference revealed no significant difference in serum levels of third complement component (C3) on days 10 and 15 compared to the PI group (Fig. 2K). Immunocytochemistry analysis of the cultured podocytes showed no evidence of any immunoreactivity with serum from APA-treated mice on day 10.

Surprisingly, 10 days after podocyte transplantation (PT), proteinuria significantly decreased in the cell transplanted anti-podocyte nephropathy induced (APN + PT) group (0.393 ± 0.07 mg/dl) compared to the PBS treated anti-podocyte nephropathy induced (APN + PBS) group (0.95 ± 0.16 mg/dl). The urine albumin/creatinine ratio also significantly decreased in the APN + PT group (1447.81 ± 231.07 µg/mg) compared to the APN + PBS group (2571 ± 347.78 µg/mg), 25 days after PT. No significant changes observed at these levels until day 50 after transplantation (Fig. 2B,C).

We observed significantly higher serum total protein and albumin levels compared to the APN + PBS group after transplantation of the cells (Fig. 2D,E). There were decreased levels of serum urea nitrogen, triglycerides, and cholesterol by the time in the podocyte-transplanted groups (Fig. 2F–H). In contrast, no significant change was observed in urea content of the urine samples during the entire experiment in any of these groups (Fig. 2I). Of note, the increased serum creatinine levels did not change up to day 50, while serum creatinine decreased on day 60 in the podocyte-transplanted groups (Fig. 2J).

We also evaluated proteinuria by SDS-PAGE of the urine samples from PI, APN + PBS, and APN + PT groups. The urine protein content decreased in the APN + PT group compared to the nephrotic mice from the APN + PBS group (Fig. 2L). Western blot analysis of proteinuria in mouse urine showed the presence of IgG, albumin, and podocyte-specific protein content such as podocin and podocalyxin, which indicated podocyte damage within the glomeruli due to APA-induced proteinuria (Fig. 2M). Western blot analysis of the urine sample from the cell-transplanted mice also showed podocalyxin and a weak band of GFP (Fig. 2M) which indicated possible transplanted GFP^+^ podocyte damage or death.

### Renal histopathologic changes in proteinuria induced and cell-transplanted mice

Histological analyses of mice nephrotic injury on day 10 showed increased mesangial matrix associated with some degrees of crescent and diffuse mesangial sclerosis (Fig. 3A), decreased Wt1^+^ podocyte numbers (Fig. 3B,E), and increased glomerular section area (Fig. 3F), compared to the NT and PI treated mice. We observed no remarkable pathological changes in the distal and proximal tubules. In addition, no GFP^+^ cell was observed in the lung and liver, 40- and 50-day post-transplantation.

**Figure 3:** Altered histopathology of membranous nephropathy (MN) obtained from 100 glomeruli per group (n = 5) with similar staining patterns on day 10. (**A**) Hematoxylin and eosin (H&E), Masson’s trichrome (MT), and periodic acid-Schiff (PAS) stained kidney sections from non-treated (NT), preimmune antibody (PI), and anti-podocyte antibody (APA) treated mice showed increased mesangial matrix and diffuse mesangial sclerosis with an occasional tendency for glomerular crescents (asterisks). (**B**) Representative pictures for immunohistochemical (IHC) staining of Wt1 as a podocyte marker in glomeruli of the 3 mice groups. (**C**) Transmission electron microscopy (TEM) revealed podocyte vacuolization with blebbing, foot process effacement, and detachment from the GBM in APA-treated mice (arrows). (**D**) Electron microscopy showed subepithelial electron dense deposits. Immunofluorescence study results showed the presence of APA, coarse granular deposits of IgG and C3 together whit C3b. (**E**) Quantitation of the numbers of Wt1-positive podocytes in the glomeruli of the 3 mice groups. (**F**) Quantitative analysis of glomerular section areas of the 3 mice groups. All values are presented as mean ± SEM. Differences were determined by ANOVA and a subsequent Tukey test. p < 0.05 was considered statistically significant. **p < 0.01, ***p < 0.001, and ns: Not significant. Scale bars in A and B: 100 µm.

Transmission electron microscopy (TEM) analysis of tissues from mice with proteinuria showed evidence of podocyte vacuolization, blebs, foot process effacement, and detachment from the glomerular basement membrane (GBM) compared with the control groups (Fig. 3C). TEM also revealed subepithelial electron dense deposits. Immunofluorescence exhibited the presence of APA, coarse granular deposits of IgG, C3, and C3b into glomerular tuft (Fig. 3D), whereas control mice did not show IgG reactivity and C3 deposition (Supplementary Fig. S5). In contrast, C1q and C4b, as the complement components, were not detected within the glomeruli.

We sought to determine if iPSC-PT has a beneficial effect on regeneration or repair after APN. Since the earliest time point at which a significant decrease in proteinuria was observed, was day 20, the mice were sacrificed on days 20, 50, and 60 and we conducted histological investigations of their renal tissues. Light microscopy assessment showed no significant pathological changes in the proximal and distal tubules throughout the observation period. The injected cells were mainly located in the cortex; however, these cells were also scattered throughout the medulla sections of the transplanted mice and occasionally in the cortical tubules (Supplementary Fig. S6). Ten days after the iPSC-PT, there were significant changes in the glomeruli that remained for an additional 40 days. We observed a significant improvement in glomerular pathologies in the podocyte-transplanted mice (Figs 4 and 5A,B). These beneficial effects were associated with a significant decrease in glomerular section area (µ^2^) in the cell-treated groups (similar to the PI-treated mice) compared to the APN + PBS groups throughout the experimental period. The glomerular section area on day 50 in these groups was 968.7 ± 36 µ^2^ for APN + PT, 1238.35 ± 39 µ^2^ for APN + PBS, and 1049 ± 33.2 µ^2^ for PI. On day 60, it was 1052.2 ± 42.1 µ^2^ for APN + PT, 1195 ± 38.8 µ^2^ for APN + PBS, and 1007.5 ± 33.2 µ^2^ for PI as seen in Fig. 5C. Immunohistological (IHC) studies of the kidney sections demonstrated that the number of Wt1^+^ podocytes decreased by approximately 50% in APA (13.2 ± 0.4) compared to PI treated (25.3 ± 0.7) mice on day 10 (Fig. 3E). The podocyte population was 17 ± 0.8 (APN + PBS) compared to 24.8 ± 0.9 (PI) on day 60 (Fig. 5D). It seems that almost 4 podocytes were ineffectively regenerated by possible renal progenitor cells until the end of the experiment. Interestingly, there was a significant increase in the glomerular podocyte population in the APN + PT groups compared to the APN + PBS groups throughout the experimental period (Supplementary Table S4).

**Figure 4:** Histopathology section of kidney specimens obtained from anti-podocyte nephropathy + phosphate-buffered saline (APN + PBS), preimmune antibody (PI), and podocyte transplantation (APN + PT) groups on days 20, 50, and 60. Representative images show hematoxylin and eosin (H&E), Masson’s trichrome (MT), and periodic acid-Schiff (PAS) staining of the kidney sections. The arrows indicate increased mesangial matrix, diffuse mesangial sclerosis with some degrees of crescent formation in the anti-podocyte nephropathy + phosphate-buffered saline (APN + PBS) groups (vehicle) compared to the preimmune antibody (PI) groups (control groups). In contrast, the representative images show significant improvement against damaged glomeruli of the cell-transplanted groups (APN + PT) compared to vehicle groups on the respective days. Scale bars: 100 µm.

**Figure 5:** Attenuation of podocyte lesion-related histological damage after induced pluripotent stem cell-podocyte transplantation (iPSC-PT) into mice with membranous nephropathy. (**A**,**B**) Percentages of glomerular pathologies; (**C**) glomerular section areas; (**D**) the numbers of Wt1-positive cells in the glomeruli of the 3 groups: preimmune antibody (PI), anti-podocyte nephropathy + phosphate-buffered saline (APN + PBS), and podocyte transplantation (APN + PT) on the indicated days.

The Wt1^+^ podocyte numbers on day 20 were 24.1 ± 0.9 (APN + PT), 14.4 ± 0.8 (APN + PBS), and 25.4 ± 0.7 (PI). On day 50, these values were 21.5 ± 0.8 (APN + PT), 16.1 ± 0.7 (APN + PBS), and 23.7 ± 0.8 (PI). On day 60, these values were 22.5 ± 0.9 (APN + PT), 17 ± 0.8 (APN + PBS), and 24.8 ± 0.8 (PI) as seen in Fig. 5D. However, in the cell-transplanted mice, the highest number of GFP^+^ iPSC-podocytes localized in the glomeruli 10 days after transplantation (9.8 ± 0.5 GFP^+^ podocyte/glo. sec. area) followed by 8.2 ± 0.4 GFP^+^ podocyte/glo. sec. area (day 40 of PT), and 7.1 ± 0.3 GFP^+^ podocyte/glo. sec. area (day 50 of PT; Fig. 6A,B). Finally, immunogold staining confirmed the incorporation of GFP^+^ podocytes in the glomeruli with apicobasal polarity and formation of SD-like structures between the FPs of newly integrated podocytes (Fig. 6C).

**Figure 6:** Qualitative and quantitative analysis of localization of transplanted podocytes. (**A**) Immunohistochemical (IHC) staining for localization of green fluorescent protein (GFP)^+^ positive transplanted induced pluripotent stem cell (iPSC)-podocytes in glomeruli 10, 40, and 50 days after cell transplantation. The maximum glomerular localization was observed 10 days after transplantation and continued up to day 50. In addition, the number of extraglomerular transplanted podocytes decreased over time. Scale bars: 100 µm. (**B**) Quantitation of the numbers of GFP^+^ iPSC-podocytes localized in the glomeruli. (**C**) Representative image of immunogold labelling confirmed the incorporation of GFP^+^ podocytes in glomeruli with apicobasal polarity and formation of slit diaphragm-like structures (arrows) between the foot processes of newly integrated podocytes, 10 days after transplantation. Scale bars: left panel: 5 µm, right panels: 500 nm. Data obtained from 100 glomeruli per group (n = 5 per group). All values are presented as mean ± SEM. Differences were determined by ANOVA and a subsequent Tukey test with p < 0.05 considered statistically significant. *p < 0.05; **p < 0.01; ***p < 0.001; and ns: Not significant.

## Discussion

Recent experiments have demonstrated that cell-based therapy as a novel strategy is potentially a promising approach for treatment of the kidney diseases or slowing its progression. Thus, in this field, cell therapy currently focuses on preclinical studies. Preclinical investigations have revealed beneficial effects of various stem cells and stem cell-derived cells in acute/chronic kidney injury models, suggesting a renal regenerative effect for the cell-based therapies^39^. Among various candidates, iPSCs have shown promising therapeutic potential for kidney disorders^40–42^. This is supported by several studies demonstrating the differentiation of iPSCs into renal lineage^20,34,43,44^ and organoids^45,46^ as well as their capabilities for *in-vivo* transplantation^47,48^ and generating complex kidney structures^49,50^.

There is a growing interest in stem cells’ differentiation into defined renal cells such as tubular^31,51^ and podocyte cells^20,22,24,34,52^. Despite reports on the therapeutic effects of iPSC-derived podocytes in experimental models^26,53^, no investigation has evaluated the potential therapeutic effects of iPSC-podocytes in an animal model of immune-mediated podocyte injury.

To this end, we generated an experimental model of MN^5,54^ by injection of rabbit polyclonal APA into mice which led to direct antibody-mediated damage of podocytes^55,56^. This model setting exhibited proteinuria associated with GBM disruption, podocyte FPs effacement, subepithelial electron dense deposits that quite closely recapitulates the morphologic hallmarks of human MN. While our serum analysis showed no significant difference in serum levels of C3 our stainings showed deposition of IgG, C3, and C3b on glomeruli together with rabbit polyclonal APA. It is assumed that based on our negative results for C1q and C4b, glomerular injury could possibly be mediated by other mechanisms than complement or at least not via the classical pathway^55,56^.

Thereafter, we developed a 3-stage protocol to obtain functional podocytes from proteinuria-induced mouse iPSCs which were evaluated with respect to constitutive and induced expression of podocyte markers. We initially used a previously reported protocol^29^ optimized for inducing the differentiation of NIM cells from mouse iPSCs. This protocol used a combination of activin A, CHIR99021 (glycogen synthase kinase 3β inhibitor), and TTNPB (pan retinoic acid receptor agonist) followed by combined treatment with bone morphogenetic protein (BMP)7, recombinant mouse leukemia inhibitory factor (mLIF), and TTNPB. The induced NIM cells expressed Osr1, Pax2, and Sall1 in conjunction with other NIM markers*, Lhx1, Eya1*, and *Wt1*^57^. NIM cells were subsequently differentiated into NPCs by treatment with BMP7, mLIF, and GDNF that expressed the specific transcription factors *Six2, Hoxd11, Cited1, Pax2*, and *Wt1*^34^. The podocyte cells had typical morphologic features; transcriptome expressions of Synpo, Nphs1, Pdxl, Nphs2, Wt1, and Pax2; and proteins (nephrin, synaptopodin, podocin, podocalyxin, and Wt1) – all essential, well-described markers of podocytes^58^ as well as actin cytoskeleton, as an important part of the podocyte-GBM interaction^59^. They also lost proliferative capacity at passage 6 exhibiting key podocyte phenotypes such as actin reorganization upon insulin or AII stimulation and albumin uptake. The protocol established in this study to differentiate iPSCs into podocytes was approximately 80% efficient in the presence of podocin as a podocyte marker protein.

Next, iPSC-derived cell suspension was slowly injected into different sites of the renal cortex parenchyma of APN-induced mice and relative improvements in renal function and critical amelioration of glomerular defects were observed. The immunohistochemical and immunogold electron microscopy analyses showed integration of GFP^+^ podocytes in glomeruli with apicobasal polarity, and formation of FPs and SD-like structures suggesting their contribution to reconstruction of the injured filtration barrier. According to our results, it is tempting to speculate that injured glomeruli could possibly provide a molecular recognition sink for transplanted iPSC-podocytes to migrate and incorporate into the injured glomeruli^60^. This result is also consistent with previous reports showing the integration of podocytes with glomeruli, indicating their capability in regeneration of injured renal structure and function^19,26^.

Although injected cells were mainly distributed in the cortex, they exhibited a scattered distribution pattern in the medulla sections and were occasionally found in the cortical tubules; however, they were not observed in the lung and liver, as the main organs of the vascular system. This finding might be attributed to the existence of differentiated tubular cells in injected cell population and also dedifferentiation of not-integrated iPSC-podocytes into tubular and/or other cells leading to their distribution in non-glomerular areas. We did not observe remarkable pathological changes in the examined areas; however, dedifferentiation of transplanted iPSC-podocytes and characterization of iPSC-non-podocyte cells should be investigated in further studies to explain the present findings.

On the other hand, we observed the presence of podocalyxin and GFP in the urine of mice during the post-transplantation period. This finding indicated possible damage or death of the transplanted GFP^+^ podocytes that led to reductions in the number of transplanted cells over time. This observation could be attributed to the rigors such as mechanical stress during implantation, extracellular matrix loss upon delivery, nutrient and oxygen deprivation at the recipient site, and host inflammatory response which are detrimental factors that limit long-term survival of transplanted cells^61–63^. Of note, the majority of regenerated podocytes in the treated APN mice, was originated from the transplanted cells, which suggested that purified iPSC-podocytes transplanted by an improved approach, might enhance the therapeutic efficacy of transplanted cells. The remainder of the regenerated podocytes might be induced by differentiation of the putative progenitor cells derived from the glomerular parietal epithelium of Bowman’s capsule^64^, which likely occurred via triggering Notch^65^ and Wnt-β-catenin pathways^66^. Therefore, accumulating evidence points to the attenuation effect of transplanted cells on proteinuria. We propose this effect is related to integration and replacement of transplanted cells and to some extent, the recruitment of intrinsic glomerular progenitors in responses to damages to podocyte pathways. Further work is required for characterization of nonintegrated cells and development of strategies that aim at improvement of viable cell engraftment and survival. Finally, it should be noted that generalization of the results of this study to human disease requires further studies to solve above mentioned limitations.

## Conclusions

We demonstrated that the transplanted iPSC-podocytes could restore injured kidney function and improve pathological indices in an experimental model of MN. These findings suggested that autologous and patient-specific iPSC-podocytes (potentially with correction of defective genes) could be a potential cellular resource for stem cell-based therapy for MN and hereditary forms of CKD. Finally, it could be an initial pace to navigate a therapeutic approach for individuals who suffer from CKD due to loss of podocytes.

## Methods

### Animal procedures and cell culture

All animal care, including experimental, surgical, and postoperative euthanasia procedures were performed in strict accordance with the ethical principles of the NIH Guide for the Care and Use of Laboratory Animals and approval by the Institutional Review Board and Ethical Committee at Royan Institute (No. EC.89.1061). Supplementary information provides more details on animal procedures, and podocyte and mesangial cell line culture protocol.

### Anti-podocyte antibody (APA) production, purification, and characterization

Rabbit polyclonal antibody against murine podocytes was generated, purified, and characterized as previously described with few modifications (Supplementary information).

### Generation of a mouse model of membranous nephropathy

This procedure was carried out as previously described with few modifications. Briefly, the animals received intravenous (IV) administration of APA 5 days after subcutaneous pre-immunization. Then, urine, serum, and tissue samples were collected (Supplementary information).

### iPSCs generation and characterization

iPSCs were derived from induced APN mouse TTFs by retroviral transfection of *Oct4*, *Sox2*, *Klf4*, and c-Myc (Addgene) as previously described (Supplementary information).

### iPSCs differentiation into podocytes

We converted the iPSCs into podocytes via a series of modified differentiation procedures to obtain stage-specific cell types of NIM, NPC, podocyte progenitors, and podocytes (Supplementary information).

### Cell proliferation assay

On day 22 of the differentiation protocol, iPSC-podocytes were seeded in 4-well plates at approximately 40% confluency. We determined the proliferation rate, expressed as doubling times, by fitting the % phase object confluence data points between day 0 to the day when cells reached 80% confluency for the next subcultures. The subcultures were continued until the cells exhibited a growth arrest. Undifferentiated E11 cells were cultured as a control group.

### Functional assays

Functional assays for iPSC-podocytes included the reorganization of F-actin cytoskeleton and contractile response to the addition of insulin (100 nM) and AII (500 nM), and the endocytosis of albumin (Supplementary information).

### Cell transplantation

We transplanted passage-6 iPSC-cells into the renal cortex parenchyma by a micropipette connected to a microinjector, 10 days after antibody treatment (Supplementary Fig. S7). The control group received PBS injections (Supplementary information).

### Evaluation of urine, serum, and histopathological indices

Supplementary information provides details on urine, serum, and histopathologic analyses and quantification of podocyte numbers.

### Statistical analysis

Values represent mean ± standard error of mean (SEM). Analysis was performed using GraphPad Prism 6.01. Differences among the experimental groups were tested by means of two-way analysis of variance with the Tukey multiple comparison test. The independent sample student’s t-tests were performed to identify significant differences in serum levels of the C3 value of the control and day 10 or 15, as well as differences in podocyte numbers at the indicated times. Statistical significance was set at p < 0.05.

## Supplementary information

Supplemental information

Supplemental movie 1

## Data Availability

The data that support the findings of this study are available from the corresponding author upon reasonable request.
